The article "An Efficient Classification of Neonates Cry Using Extreme Gradient Boosting-Assisted Grouped-Support-Vector Network" was published in 2021. Journal: J Healthc Eng.

# An Efficient Classification of Neonates Cry Using Extreme Gradient Boosting-Assisted Grouped-Support-Vector Network

**DOI:** 10.1155/2021/7517313

**Published:** 2021-11-11

**Authors:** Chuan-Yu Chang, Sweta Bhattacharya, P. M. Durai Raj Vincent, Kuruva Lakshmanna, Kathiravan Srinivasan

**Affiliations:** ^1^Department of Computer Science and Information Engineering, National Yunlin University of Science and Technology, Taiwan; ^2^Service Systems Technology Center, Industrial Technology Research Institute, Hsinchu, Taiwan; ^3^School of Information Technology and Engineering, Vellore Institute of Technology, Vellore 632 014, Tamil Nadu, India; ^4^School of Computer Science and Engineering, Vellore Institute of Technology, Vellore 632 014, Tamil Nadu, India

## Abstract

The cry is a loud, high pitched verbal communication of infants. The very high fundamental frequency and resonance frequency characterize a neonatal infant cry having certain sudden variations. Furthermore, in a tiny duration solitary utterance, the cry signal also possesses both voiced and unvoiced features. Mostly, infants communicate with their caretakers through cries, and sometimes, it becomes difficult for the caretakers to comprehend the reason behind the newborn infant cry. As a result, this research proposes a novel work for classifying the newborn infant cries under three groups such as hunger, sleep, and discomfort. For each crying frame, twelve features get extracted through acoustic feature engineering, and the variable selection using random forests was used for selecting the highly discriminative features among the twelve time and frequency domain features. Subsequently, the extreme gradient boosting-powered grouped-support-vector network is deployed for neonate cry classification. The empirical results show that the proposed method could effectively classify the neonate cries under three different groups. The finest experimental results showed a mean accuracy of around 91% for most scenarios, and this exhibits the potential of the proposed extreme gradient boosting-powered grouped-support-vector network in neonate cry classification. Also, the proposed method has a fast recognition rate of 27 seconds in the identification of these emotional cries.

## 1. Introduction

Crying is the primary mode of communication among infants to make their care givers aware of their physiological and psychological necessities. It is also the first expression of life at birth. The reasons behind infant crying can be numerous. A crying infant achieves the objective of attracting attention of the caregiver informing that the baby needs an interaction of some sort. Infant cries hold enormous information on its sound wave, and often the sound provides insight on the reason and severity of the cry. Infant cry is an important indicator of various types of information–emotion, gender, maturity at birth, first cry, and health status, and sleep pattern of the infant. The activity of crying is controlled by the brain and is triggered in case of any exceptional event occurring against the normal functioning of the infant's body. It acts like an alarm to inform on any alternated event pertinent to the functioning of the body, being reflected as a cry. The event of crying encompasses sequences of motor skill performances along with acoustic expressions such as vocalization, coughing-choking, constrictive silence, and various combinations of these manifestations.

The article "An Efficient Classification of Neonates Cry Using Extreme Gradient Boosting-Assisted Grouped-Support-Vector Network" was published in 2021. Journal: J Healthc Eng.

Babies who are born before the 37 weeks of gestational period are preterm. Neonates are newborn babies born full term completing the gestational period. It is obvious that preterm babies are susceptible to various health issues and need immense care during the early developmental stage. Neonates similarly need care to ensure that growth is normal, and chances of health complications are eliminated to the maximum level. The pitch of cry in preterm and neonates contributes significantly in analyzing the signs of the problem to take immediate remedial steps at the earliest. Especially, in preterm, the sound and frequency of cry provide early information with deeper problems in comparison to other diagnostic tests, wherein pathological diseases in infants take almost seven months to a year time frame to get detected. Early detection of these diseases provides opportunities for versatile treatment applications and medical therapies. An infant cry wave contains information on the physical state and physical pathologies of babies. Processing of this information is similar to the task of pattern recognition, possessing high potential as a noninvasive complementary tool for detection and strategizing preventive steps for infant health issues.  Figure 1 depicts the waveform and spectrogram of an infant cry. Figures 2–4 illustrate the waveforms and spectrograms of sleep, hunger, and discomfort cries, respectively.

It becomes pertinent to mention that infant cries belong to the most sensitive range of human auditory sensation. Infant cries are initiated from events occurring in the respiratory and nervous system. The sound is generated from the vocal cord and vocal tract with a frequency range of 250 Hz. to 600 Hz. The first shrill cry provides significant information on APGAR count to categorize if a newborn baby could be considered as health, weak or sick. The vocalizations, time variance, and limb movements associated with infant cry provide insight on their neurological aspects. Analysis of this sound as already mentioned is important in the detection of health hazards, and various studies have been conducted in the similar direction. Originally, sound spectrogram was used as the primary tool for the analysis of crying sounds in the years 1960s and 1970s. Spectrogram was an analog device that plotted time on the *x* axis, frequency on the *y* axis, and the frequency was depicted by dark lines. The progression of the technology led to the present day use of pitch frequency, cross-correlation, Mel frequency, cepstral coefficients, and various automatic classification methodologies. These traditional methodologies emphasized on analyzing infant cry sounds based on features derived from fundamental frequency contours, pitch contours, and signal energy in different frequency subbands and unvoicing. Moreover, the frequency of crying and formants of the cry signals has been analyzed. Attempts have been made to classify infant cries based on the root causes–pain, sadness, hunger, and fear. The characteristics of the cry signal pitches have categorized cry signals as urgent, sick, and various others. Pitch detection algorithms have been implemented to calculate the instantaneous fundamental frequency (F0), wherein the first three formants along with F_0_ have been used to analyze the sounds. Machine learning enables systems to automatically learn and build the analytical model from their experience. [1–14] The work in [15] presented an extensive review of research done focusing on the analysis and classification of infant crises. The review was conducted targeting various aspects such as data acquisition techniques, cross-domain signal processing techniques, and various machine learning classification techniques. The contribution of preprocessing techniques in describing diversified features, namely, Mel-Frequency Cepstral Coefficients (MFCC), spectrogram, and fundamental frequency, is discussed. It is observed that acoustic and prosodic features that are extracted from various domains have the potential to segregate frame-based signals from one another and thus are used for the training of machine learning classifiers. The study discusses traditional machine learning techniques along with newly generated deep learning architectures and highlights future directions of research in data processing, feature extraction, and neural networks for understanding, interpreting, and processing infant cry signals.

The article "An Efficient Classification of Neonates Cry Using Extreme Gradient Boosting-Assisted Grouped-Support-Vector Network" was published in 2021. Journal: J Healthc Eng.

Although various studies have been conducted on infant cry data analysis, they lag a comprehensive methodology for the analysis and recognition of signals to achieve optimized decision making. The unique contribution of the present study involves the following:

1. Conducting exhaustive preprocessing includes seven steps, namely, standardization through normalization, framing, detection or end-point detection or cry unit, preemphasizing, windowing, and Fast Fourier Transformation.
2. Features were extracted using acoustic feature engineering, and variable selection using random forests (VSURF) was used for selecting the highly discriminative feature set.
3. Implementation of grouped-support-vector network is for an efficient infant cry classification with a faster emotional cries recognition rate of 27 seconds.
4. The proposed model yields effective results in higher dimensional spaces and is applicable in scenarios, wherein the dimension count is larger than the sample count.
5. The implementation of boosting helps create classifiers for its ensemble by training each classifier. This is achieved through random redistribution of the training datasets through the resampling process.
6. The best experimental results exhibited a mean accuracy of about 91% for most cases, and this demonstrates the potential of the extreme gradient boosting-powered grouped-support-vector network in neonate cry classification.

The following sections of this paper are organized as follows: Section 2 presents a detailed literature review.  Section 3 illustrates the proposed methodology, Section 4 presents the results and discussions, and Section 5 provides conclusion of the study.

## 2. Literature Review

Numerous studies have been conducted pertinent to the analysis and interpretation of infant cry. Some of the significant and recent studies conducted on infant cry classification are discussed in this section.  Table 1 presents a consolidated review of techniques and challenges in infant cry classification. This section highlights some of such studies and their observations.

The study in [24] emphasized the importance of automatic recognition of infant cries to develop an application that would improve the quality of life of the infant and their parents. The study generated real-time datasets from infant cries and selected the most relevant sound attributes that affected the experimental results and helped monitor infants. The framework automatically detects instances of discomfort signals, which are common among 25 percent of infants, using machine learning techniques. The study included an ensemble technique through which low-level audio features were selected from labelled precry recordings and high level features relevant to the envelop of crying. The inclusion of precry signals helped understand infant needs better, providing the opportunity to develop superior quality of baby monitors.

The article "An Efficient Classification of Neonates Cry Using Extreme Gradient Boosting-Assisted Grouped-Support-Vector Network" was published in 2021. Journal: J Healthc Eng.

The study in [25] performed an experimental analysis using two ensemble models to classify infant cry. The two models used are a boosting ensemble of artificial networks and a boosting ensemble of support vector machines. The study highlighted the superiority of the neural network-based ensemble model in the classification of infant cry. The challenges of the study included the difficulty of collecting cry samples from normal babies without any pathology, pain, or hunger issues. The availability of a larger number of samples would help generalize the results achieved and justify the possibility of its application in real time.

There have been immense advancements in perinatology and neonatology, which have created a positive impact in the survival of preterm and low weight neonates. The study in [26] highlighted the importance of infant cry analysis as a noninvasive complementary tool for the assessment of the neurological conditions of premature neonates. The study emphasized on identifying the distinctions between full-term and preterm neonatal cry using automatic acoustical analysis in association with various data mining techniques.

The act of crying is a sole method of for infants to communicate with their environment to inform about their necessities and issues. These audio signals require thorough analysis and extraction of features with the help of expert knowledge. The use of deep learning does not require much of preprocessing and is capable of extracting important features automatically from the datasets. The study in [27] implements a deep learning-based feature extraction technique followed by machine learning algorithms for the classification of infant cry. The audio signal of 4-second duration was transformed into a spectrogram image and then fed into the DCCN for extraction of features. The extracted features were further classified using ML algorithms, namely, SVM, Naïve Bayes, and KNN. The framework was evaluated with the Bayesian hyperparameter optimization technique. The results highlighted the superiority of SVM in the classification of infant cry due to hunger, pain, or sleepiness.

The study in [28] implemented machine learning techniques to analyze distress calls among infant chimpanzees. The exemplars were extracted from the distress call episodes, and the external events that caused such calls and the distance from the mother were analyzed to identify any correlations. The results revealed that such distress calls could provide information on discrete problems faced by the infants and their distance from the mother. These factors would act as a guide for maternal decision making. However, the role of acoustic cues in this regard has remained a topic of future scope of research.

The article "An Efficient Classification of Neonates Cry Using Extreme Gradient Boosting-Assisted Grouped-Support-Vector Network" was published in 2021. Journal: J Healthc Eng.

The study of infant cry recognition helps identify the typical needs of infants from their care givers. Different cry sounds portray different meanings and help the caregivers respond appropriately, which further influence their emotional, behavioral, and relationship development. The recognition of infant cries is quite more difficult than understanding of adult speech due to the absence of verbal language-based information. The study in [29] analyzes different types of emotional necessity as communicated by infants through their cry, namely, due to hunger, sleepiness, stomachache, uneasiness, and need to burn. A combination of CNN and RNN is used for feature extraction and classification. The CNN-RNN method when implemented in the study outperforms the traditional methods in terms of accuracy up to 94.97%.

The use of IoT and smart devices has helped develop state-of-the-art infant incubators that would enable caregivers to respond quickly to the specific needs of the infants. The baby voices are classified using machine learning using the open voice database. The sensor-based incubator as proposed in the study [30] would help in reporting the infant's condition. The use of IoT technology would enhance the function of the actuators inside the incubator. Finally, the combination of historical data and the live data collected by the sensors would provide extensive information on the infant's condition and the environment.

The study in [31] used neural networks to analyze the source of infant crises. The work combined the genetic algorithms, ANN in association with linear predictive coding (LPC) and MFCC for the classification of infant cries. The results justified the superiority of the proposed method when compared with other traditional approaches.

The study in [32] used Gaussian mixture model–universal background model for the recognition and analysis of infant cry signals even when there are channel imbalances and corroded signals. The results proved to be much superior when compared with high-order spectral features ensuring enhanced accuracy.

The study in [16] highlighted the importance of explicit and relevant feature representation of infant cry signals, which are significantly different from speech signals. The study proposed the use of unsupervised auditory filterbank learning implementing convolutional restricted Boltzmann machine (ConvRBM) model. The model was able to successfully distinguish the differences between normal and pathological crying signals. The model, when compared with the mel-frequency cepstral coefficient model (MFCC), performed better in terms of accuracy. However, the model was not evaluated against any other model apart from MFCC.

The article "An Efficient Classification of Neonates Cry Using Extreme Gradient Boosting-Assisted Grouped-Support-Vector Network" was published in 2021. Journal: J Healthc Eng.

The study in [17] presented a review of various techniques adopted in infant cry analysis and classification. The reviews were primarily focused on different aspects of data acquisition, signal processing techniques across various domains and different machine learning based classification techniques. The paper discussed diversified features, namely, MFCC, fundamental frequency, and spectrograms. The study also highlighted the use of traditional machine learning models such as KNN, GMM, and SVM and latest models CNN and RNN in infant cry identification, analysis, classification, and detection. The scalability of datasets, unavailability of skilled labor for collecting data, and lack of collaboration between medical professionals and researchers were identified as the challenges in infant cry research.

The study in [18] proposed a CAD system that helped differentiate the healthy and unhealthy infant cry signals. The system constituted of four stages: firstly, the preprocessing of the cry signals was done to remove background noise and signal segmentation was carried out. Then, the preprocessed signal was analyzed to attain its cepstrum. Thirdly, the cepstrum coefficients were fed into a deep feed forward neural network (DFNN) for the purpose of training and classification. Finally, the system was evaluated against the standard classification performance metrics. The study did not include classification of deep features and nonlinear statistical features.

The study in [19] implemented convolutional neural network (CNN) for classifying the infant vocal sequences. The classes identified were, namely, “crying,” “fussing,” “babbling,” “laughing,” and “vegetative vocalization.” The audio segments were represented as spectrograms and fed into the conventional CNN. The accuracy achieved was quite balanced. The model, however, was not evaluated against any other models.

The study in [20] developed a smart cradle that operated based on the sounds of the infant. The infant sounds were classified using support vector classifier (SVC) and radial basis function (RBF) kernel based on 18 features extracted from the infant sounds. The system was evaluated against linear and polynomial SVC functions and other traditional classification models like Decision Tree, Random Forest, and Naïve Bayes algorithms. The proposed system was identified to be working with enhanced accuracy in comparison to the other traditional approaches. The study was based on only 4 types of sound, and hence, inclusion of more sound categories would help justify the accuracy of the model with enhanced accuracy.

The article "An Efficient Classification of Neonates Cry Using Extreme Gradient Boosting-Assisted Grouped-Support-Vector Network" was published in 2021. Journal: J Healthc Eng.

The study in [21] performed infant cry classification based on different features that were extracted from the processing of speech and auditory dataset. The model at the outset was trained using the individual features. Then, the most significant features were selected, and the model was retrained combining these selected features. SVM, KNN, logistic regression, and random forest models were used for the purpose of classification. The model could be further evaluated using an extensive dataset for further evaluation and justification of the proposed approach.

It was emphasized in [22] that duration and frequency of infant crying were important identifiers for child health condition. The manual monitoring and observation in this regard were extremely taxing and had possibilities of indicating erroneous results. The study thus focused on developing a smart phone-based framework to automatically detect infant crying. Datasets of infant crying clips were collected from different online sources, and the audio features were extracted from these clips using the OpenSMILE software. The random forest algorithm was used to classify the crying and noncrying audio clips, and then, the model was evaluated using real-time audio clip recordings. The Motorola G5/*G*6 phones were used for experimentation. Hence, the performance of the model in case of other smart phones remains uncertain.

The study in [23] classified infant crying sounds using the Higuchi fractal dimensions. The KNN and SVM algorithms were used for the purpose of classification. Both algorithms were evaluated, and the results revealed that SVM performed better than KNN in terms of accuracy. The study could be further improved by including more types of infant cries and an extensive dataset that would help justify the superiority in the performance of the proposed approach.

## 3. Materials and Methods

### 3.1. Preprocessing of Infant Cries and Feature Extraction

Figure 5 represents the flow diagram of the proposed neonate cries classification system.

The second step in the proposed framework involves preprocessing of the dataset, which helps in eliminating inferences and disturbances existing in the cry data. An exhaustive preprocessing is performed, which includes seven steps, namely, normalization, framing, end-point detection, cry unit detection, preemphasizing, windowing, and fast Fourier transformation. The preprocessing is succeeded by feature extraction (acoustic feature engineering), which helps eliminate irrelevant features from the dataset and consider features, which contribute significantly to the overall output of the classification.

The article "An Efficient Classification of Neonates Cry Using Extreme Gradient Boosting-Assisted Grouped-Support-Vector Network" was published in 2021. Journal: J Healthc Eng.

The classification of infant mode cries specifically by audio signals would lead to the generation of a large amount of data having difficulty in identification. Hence, the input signal is converted to a relatively concise feature vector, and the characteristic parameters are extracted, which represent the cry signal. In the case of signal analysis pertaining to the time domain without conversion, relatively lesser features are extracted from the original signal without making it damaged or lost. On the contrary, in the case of signal analysis pertinent to frequency domain, relatively more features get extracted from the original signal without much damaging or loss of the same, while the audio signal gets converted from the time domain to frequency domain. Thus, in this study, features are extracted from both time domain and frequency domain to achieve enhanced identification of infant cry models.  Table 2 lists the twelve extracted features using acoustic feature engineering.

The variables used in the study are as follows:

- *S*_*j*_(*n*): indicates the signal of the *j*-^th^ frame in the time domain
- *S*_*j*_′(*n*): indicates the signal of the *j*-^th^ frame in the frequency domain after framing, Hamming windowing, and fast Fourier transformation.
- *T*: represents the features extracted in time domain.
- *F*: represents the features extracted in the frequency domain.
- *N*: represents the number of samples in a frame.

Table 2 exhibits the details of the extracted twelve features. The particulars of every feature are summarized as given by the subsequent expressions:

#### 3.1.1. Magnitude

The magnitude of an audio signal is the measure of how distant it, regardless of direction, and its quantitative value differ from zero

(1) $$\begin{array}{c} {\text{TM}}_{j}=\sum_{i=0}^{N-1}\left|S_{j}\left(i\right)\right|. \end{array}$$

#### 3.1.2. Average

(2) $$\begin{array}{c} {\text{TA}}_{j}=\frac{1}{N}\sum_{i=0}^{N-1}\left(S_{j}\left(i\right)\right). \end{array}$$

#### 3.1.3. Variance

(3) $$\begin{array}{c} {\text{TV}}_{j}=\frac{1}{N}\sum_{i=0}^{N-1}{\left(S_{j}\left(i\right)-{\text{TA}}_{j}\right)}^{2}. \end{array}$$

#### 3.1.4. Zero Crossing Rate

The rate at which the signal changes from positive to zero to negative or vice–versa is termed as zero crossing rate. This value is immensely helpful in the recognition of audio signals, being a key feature for the classification of percussive sounds.

(4) $$\begin{array}{c} {\text{TV}}_{j}=\frac{1}{N}\sum_{i=0}^{N-1}{\left(S_{j}\left(i\right)-{\text{TA}}_{j}\right)}^{2}. \end{array}$$

#### 3.1.5. Bandwidth

Bandwidth is the difference between lower and upper frequencies in the case of continuous band of frequencies.

(5) $$\begin{array}{c} FB_{j}=\sqrt{\frac{\sum_{i=0}^{N-1}\left({\left|S_{j}^{\prime }\left(i\right)\right|}^{2}\times {\left(i-FC_{j}\right)}^{2}\right)}{\sum_{i=0}^{N-1}\left({\left|S_{j}^{\prime }\left(i\right)\right|}^{2}\right)}}. \end{array}$$

The article "An Efficient Classification of Neonates Cry Using Extreme Gradient Boosting-Assisted Grouped-Support-Vector Network" was published in 2021. Journal: J Healthc Eng.

#### 3.1.6. Peak

(6) $$\begin{array}{c} {\text{FPeak}}_{j,k}=\log\left\{\frac{1}{\alpha N}\sum_{i=0}^{\alpha N-1}S_{j,k,i}^{\prime }\right\}. \end{array}$$

#### 3.1.7. Valley

(7) $$\begin{array}{c} {\text{FValley}}_{j,k}=\log\left\{\frac{1}{\alpha N}\sum_{i=0}^{\alpha N-1}S_{j,k,N-i+1}^{\prime }\right\}. \end{array}$$

#### 3.1.8. Pitch

Pitch presents the perception of considering frequency based on low acoustic signal or high acoustic signal, which is analogous to the concept of fundamental frequency (*f*_0_). The basic methodology to measure *f*_0_ is to study the waveform in the time domain. Autocorrelation calculation was used to extract the pitch of the neonate cry signal in the present study.

#### 3.1.9. Formant

Formant is defined as the assortment of frequencies of a complex sound, in which there exists an absolute or relative maximum in the acoustic spectrum. Formants can be referred to as either a resonance or the spectral maximum generated by the resonance. The formants are usually measured as amplitude peaks in the frequency spectrum of the sound, using a spectrogram or a spectrum analyzer. The first six formants are extracted from the signal frame as per the characteristic parameter being represented as F1∼F6.

#### 3.1.10. LPCC

LPCC [27] is predominantly employed in various audio recognition applications. LPCC involves modeling of the human vocal tract using a digital all-pole filter. There exists *p* number of LPCCS, which are clustered together to establish one feature vector for a specific neonatal cry signal frame. In the present study, the factor *p* is fixed to a value 12, and the extracted twelve features are represented as LPCC_1_∼LPCC_12_.

#### 3.1.11. MFCC

In audio recognition systems, MFCC [26] is one of the best frequently adapted feature extraction techniques. Considering the frequency spectrum of the windowed neonatal cry signal frames, the feature vectors get extracted. Assuming that *p* is the order of the Mel scale spectrum, the feature vectors are attained considering the first *p-DCt* coefficients. In the present study, the factor *p* is fixed to a value 12, and the extracted twelve features are represented as MFCC_1_∼MFCC_12_.

#### 3.1.12. ΔMFCC

The objective of using ΔMFCCs involves the enhanced capability to recognize cry signals. This is achieved through a better understanding of the dynamics of the power spectrum, i.e., the trajectories of MFCCs over time.

The article "An Efficient Classification of Neonates Cry Using Extreme Gradient Boosting-Assisted Grouped-Support-Vector Network" was published in 2021. Journal: J Healthc Eng.

### 3.2. Feature Selection-Variable Selection Using Random Forests

The feature selection technique used in the present study is variable selection using random forests (VSURF), which is implemented using the “VSURF package” in R environment.

The steps involved in the VSURF algorithm are presented in this section. Firstly, the variables are ranked on the basis of their importance measurement, and unimportant ones are eliminated from consideration. Secondly, two different subsets are obtained either by considering a collection of nested RF models including selection of the most accurate variable or by introducing the sorted variables sequentially done. It is important to mention that each RF is typically built using ntree = 2000 trees. There are 12 features extracted in each frame. It becomes cumbersome and time consuming to use the 12 features directly to train a classifier. Hence, to reduce the computational time, the selection of discriminative features is necessary to achieve the optimum level of accuracy. As part of this study, five discriminative features, namely, peak, pitch, MFCCs, ΔMFCCs, and LPCC, are selected, which would be used as features while training the cry signals.

### 3.3. Grouped-Support-Vector Network

Support vector machines (SVMs) are a set of supervised learning methods, which are used for classification, regression, and outliers' detection in the n-dimensional hyperspace. The benefits of SVMs include its ability to perform effectively in high dimensional spaces and in cases where the numbers of dimensions are greater than the number of samples. Another significant advantage is that it deploys a subset of training points in the decision function termed as support vectors, making it memory efficient. Furthermore, SVMs can simultaneously minimize estimation errors and model dimensions. The experimental analyses were implemented in R open source platform. The SVM models in this work were devised by employing the “e1071 package” in the R library. Moreover, the major advantage of using this library is that it permits the alternation of the traditional SVM classification model and makes it possible to be implemented for the multiclass classification. For augmenting the computational speed, the “doMC package” and “foreach package” were used to permit the parallel development of the modules in the grouped model. The “doMC package” is a “parallel backend” for the “foreach package.” It presents the technique required to execute “foreach” loops in parallel. The “foreach package” delivers a new looping construct for the execution of R code repeatedly. Moreover, the “foreach package” was deployed in combination with a package named “doMC,” which would enable the code to be executed in parallel. The main objective behind the use of “foreach package” is its ability to support parallel execution, in the sense that it can execute such repeated operations on multiple cores on the workstation. Besides, by using “foreach,” this operation was executed in parallel on multiple cores, reducing the execution time back down to minutes. Furthermore, it can be witnessed that the final classification outcome of the grouped classifier is the amalgamation of the prediction of the individual classifiers. Another vital point to note is that the individual SVM classification members are diverse, and they also have precise and unique performance, which makes it easier for the grouped-support-vector network to have a more accurate prediction.  Figure 6 shows the infant cry classification using grouped-support-vector network.

The article "An Efficient Classification of Neonates Cry Using Extreme Gradient Boosting-Assisted Grouped-Support-Vector Network" was published in 2021. Journal: J Healthc Eng.

### 3.4. Boosting

Bootstrapping, which is also known as bagging, is a predominantly used sampling technique. It is an ensemble method that creates classifiers to implement an ensemble approach. This is achieved by training each of the classifiers, following a random redistribution of the training datasets using the resampling technique. It thus incorporates the best of both bootstrap and aggregating techniques. In case of boosting, “r” samples are chosen out of the “p” available samples with replacement. The learning algorithm is then implemented on each of these samples. The point of sampling with replacement is to ensure that the resampling performed is random in the truest sense. If the point of sampling is performed without replacement, the samples drawn would be dependent on the previous ones and hence will not be random. The predictions from the above models are aggregated to conclude to the final combined predictions. The aggregation could be done on the basis of predictions made or the probability of the predictions made by the individual bootstrapped models. The random sampling method based on the bagging technique is applied repeatedly to attain a group of member classifiers.

The use of bagging in resampling of the training subset using bootstrapping of each classifier within the ensemble helps achieve diversity. In such circumstances, a dissimilar training subset is extracted from the original training set using the technique “resampling with replacement,” thereby generating “m” number of subsets. Each one of these generated subsets is further used to train a classifier within the ensemble. This developed ensemble further used helps predict a subset of unseen testing data, wherein the output of the classifiers inside the ensemble is combined using weighted majority voting. In case the ensemble classifier fails to get similar prediction accuracy, providing more voting weight to the classifier having high accuracy is considered the best fit. This approach is known as weighted majority voting. Combining bootstrapping with the weighted majority voting aggregation method leads to the development of a new category of ensemble-based systems called “boosting.” The objective is to assign higher “weights” to classifiers, which have high accuracy during the training process, whereas assigning lower weights to classifiers has lower accuracy, which would increase the probability of correct final output of the ensemble model.

The article "An Efficient Classification of Neonates Cry Using Extreme Gradient Boosting-Assisted Grouped-Support-Vector Network" was published in 2021. Journal: J Healthc Eng.

Extreme gradient boosting (XGBoost) is implemented using the “xgboost package.” It is a scalable and efficient application of gradient boosting framework, which helps perform parallel computation automatically. In XGBoost, the decision trees are developed in sequential form. The weights take an essential role in XGBoost being assigned to the independent variables. It is fed to the decision tree, which helps in predicting the results. In case the weight of the variables is predicted inaccurately by the tree, the respective value is increased, and further, variables are fed into a second decision tree. These individual classifiers are then combined or ensemble to develop a stronger and more accurate model. The ensemble SVM model is initially optimized by identifying the best regularization parameter “C” for the training criterion and the bandwidth “*γ*” for the Gaussian kernel. For the sake of achieving the same, a grid search is implemented using the parameters “C” = [1,3,33] and “*γ*” = [0.1, 0.2, 0.3,., 5]. The entire dataset TR is first segregated into training TR_*m*_ and testing subset VA_*m*_ as per 80 : 20 ratio, respectively. The radial basis function (RBF) kernel is used in the development of SVM regression models. The final SVM classifier is then developed using these parameters before being added to the ensemble. This procedure is repeated 300 times until the entire ensemble is generated. The final ensemble classification is finally calculated using a weighted majority voting approach.

## 4. Results and Discussion

Figure 7 illustrates the infant cry acquisition setup. The dataset used in this study consisted of 258 sleepy cries, 372 hunger cries, and 372 discomfort cries taken from 12 female and 17 male infants having an age between one to ten days. These newborn babies were located at the department of Obstetrics and Gynecology, National Taiwan University Hospital Yunlin Branch, Taiwan. Additionally, the newborn babies were normal and had no pathological background. Moreover, these infant cries were classified into three categories, namely, sleepy, hunger, and pain-induced cries. During the acquisition of the cry, the infants were placed in the semisupine position: the infants facing upward with their head resting on a cradle and their neck in a neutral position. The infant's arms were in a neutral thumb position. Sony HDR-PJ10 High Definition Camcorder was deployed to record the infant cries with a 44.1 kHz sampling rate of 16 bits of resolution. The distance between the infant's mouth and the camcorder microphone was around 40 cm. The lengths of recorded infant cries were between 10 and 60 seconds. The infant cry measurement setup is illustrated in Figure 7. This research was approved and accepted by the ethical review committee from the National Cheng Kung University Human Research Ethics Committee. The parents of the infants had provided their written consensus for being a part of this study. All experimental results were validated using 10-fold cross-validation. The benefit of this process is that, during the training and validation, it completely includes all the data samples; however, a data sample is deployed only once for validation purposes.  Table 3 lists the dataset deployed for training and testing purposes.

The article "An Efficient Classification of Neonates Cry Using Extreme Gradient Boosting-Assisted Grouped-Support-Vector Network" was published in 2021. Journal: J Healthc Eng.

### 4.1. Infant Cry Classification Based on the 12 Extracted Features

The twelve extracted features were deployed in the experiment. Among all considered cry signals, eighty percent of the cry signals were employed in training, and twenty percent were utilized for testing.  Table 3 collates the number of cries deployed in the training and testing of the dataset. There are totally 372 hunger cries, 258 sleep cries, and 372 discomfort cries.  Table 4 presents the classification accuracy based on the extracted 12 features. It can be observed that the mean cry classification accuracy is around 91 percent. Further, the discomfort cries have the highest classification accuracy of 95 percent.  Figure 8 portrays the receiver operating characteristic curve of the proposed model with 12 features.

The accuracy can be computed from the following expression:

(8) $$\begin{array}{c} \text{accuracy}=\;\frac{\text{number of correctly predicted cries}}{\text{total number of cry predictions}}. \end{array}$$

### 4.2. Infant Cry Classification Based on the Selected 5 Features

In this experiment, the dataset exemplified in Table 2 was employed.  Table 5 describes the confusion matrix for the infant cry classification based on the selected 5 features, namely, Peak, Pitch, MFCCs, ΔMFCCs, and LPCC. Further, the discomfort cries have the highest classification accuracy of 96 percent, and the mean cry classification accuracy is around 95 percent.  Figure 9 portrays the graphical representation of the classification accuracy with and without feature selection.  Figure 10 depicts the receiver operating characteristic curve of the proposed model with 5 features.

The article "An Efficient Classification of Neonates Cry Using Extreme Gradient Boosting-Assisted Grouped-Support-Vector Network" was published in 2021. Journal: J Healthc Eng.

### 4.3. Comparison of Infant Cry Classification between Male and Female Babies

In experiment 3, the classification scenario of experiment 2 is deployed for understanding the variation in cries between male and female infants. An aggregate of 422 cries comprising of 193 male and 229 female infant cries was tested in this research. The classification accuracy for distinct genders is displayed in Table 6. The classification accuracies for male and female infant cries are 93.78% and 96.19%, respectively. It can be observed that the female neonate cries have a higher accuracy than the male neonate cries.

### 4.4. Comparison of the Proposed System with Other Models

Table 7 indicates the comparison of the proposed model with the other models for different infant cry datasets. It can be witnessed that the proposed grouped-support-vector network provides better mean classification accuracy than Chang et al. [36] for hunger, sleep cry, and discomfort emotional cries. It could be witnessed that when there is a clear margin of separation between the emotional cry classes, the proposed extreme gradient boosting-powered grouped-support-vector network works excellently and is very effective in high dimensional spaces.

## 5. Conclusion

We studied numerous details about infants using newborn cry signals. Quite a few researches were found in the literature for infant classification using different approaches. This research proposed an extreme gradient boosting-powered grouped-support-vector network for infant cry classification with mean accuracy about 91% for the majority of the experimental scenarios. Initially, 12 features were extracted using acoustic feature engineering, and the variable selection using random forests (VSURF) is used for selecting the highly discriminative features. The dataset used in this study comprised 258 sleepy cries, 372 hunger cries, and 372 discomfort cries taken from 12 female and 17 male infants having an age between one to ten days. The newborn babies were normal and had no pathological background. The empirical results show that the proposed method provides a mean classification accuracy of around 91%, and this approach effectively studies even the elusive changes in the neonate cry signals with a faster recognition rate of 27 seconds. Even though the proposed method performs reasonably well for neonate cries with minimal noise, however, the performance of this system could be held back for cries with high noise levels. Therefore, in the present dataset, the unwanted noise signals were removed during the preprocessing stage. For future work, we are planning to deploy advanced deep learning and optimization approaches for achieving an improved performance.

The article "An Efficient Classification of Neonates Cry Using Extreme Gradient Boosting-Assisted Grouped-Support-Vector Network" was published in 2021. Journal: J Healthc Eng.

## Figures and Tables

**Figure 1:** Waveform and spectrogram of an infant cry.

**Figure 2:** Waveform and spectrogram of sleep cry.

**Figure 3:** Waveform and spectrogram of hunger cry.

**Figure 4:** Waveform and spectrogram of discomfort cry.

**Figure 5:** Flow diagram of the proposed system.

**Figure 6:** Infant cry classification-grouped-support-vector network.

**Figure 7:** Infant cry acquisition setup.

**Figure 8:** Receiver operating characteristic curve of the proposed model with 12 features.

**Figure 9:** Classification accuracy with and without feature selection.

**Figure 10:** Receiver operating characteristic curve of the proposed model with 5 features.

**Table 1:** Consolidated review of techniques and challenges in infant cry classification.

Ref. No.	Dataset	Methodology	Research challenges
[16]	DA-IICT infant cry and baby Chillanto	Convolutional restricted Boltzmann machine (ConvRBM) model	(i) Model was not implemented in any real-time environment (ii) Model was not evaluated against any other model apart from MFCC
[17]	Self-recorded datasets, baby Chillanto, National Taiwan University Hospital, Dunstan baby, iCOPE, University of Milano Bicocca	MFCC, KNN, SVM, GMM, CNN and RNN	(i) Scalability of the dataset (ii) Unavailability of skilled labors to collect data (iiii) Lack of collaboration between medical professionals and researchers
[18]	Sainte-Justine Hospital (Montreal, Canada), Al-Sahel Hospital (Lebanon), Al-Raee Hospital (Lebanon)	DFNN	(i) Exclusion of various topologies and transfer functions (ii) exclusion of deep features and nonlinear statistical features
[19]	Audio recordings from free sound, BigSoundBank, sound archive, ZapSplat, SoundBible and sound jay	CNN	(i) Model was not evaluated against any other models
[20]	Self-recorded audio recordings	SVC and RBF	(i) Exclusion of more features or categories in the dataset
[21]	Donate-a-cry corpus	SVM, random forest, logistic regression, KNN	(i) Exclusion of a more extensive dataset for enhanced justification of the model
[22]	Datasets from various online resources with infant cry clips	Random forest classification model	(i) Use of smart phones other than Motorola G5/*G*6 not included for evaluation
[23]	Donate-a-cry corpus	KNN and SVM	(i) Exclusion of an extensive dataset with more infant cry categories

**Table 2:** Twelve extracted features of acoustic feature engineering.

Time domain		Frequency domain	
1	Magnitude	**1**	Pitch
2	Average	**2**	Bandwidth
3	Variance	**3**	Peak
4	Zero crossing rate	**4**	Valley
		**5**	Formant
		**6**	LPCC
		**7**	MFCC
		**8**	ΔMFCC

The article "An Efficient Classification of Neonates Cry Using Extreme Gradient Boosting-Assisted Grouped-Support-Vector Network" was published in 2021. Journal: J Healthc Eng.

**Table 3:** Dataset for training and testing.

	Training data	Testing data	Total
Hunger	186 cries	186 cries	372 cries
Sleep	129 cries	129 cries	258 cries
Discomfort	186 cries	186 cries	372cries

**Table 4:** Classification accuracy based on the extracted 12 features.

System classification	Actual Classification			
	Hunger	Sleep	Discomfort	Accuracy
Hunger	168	3	15	0.9032
Sleep	7	113	9	0.8759
Discomfort	7	1	178	0.9569
Mean				0.9120

**Table 5:** Classification accuracy deploying the selected 5 features.

Actual classification	System classification			
	Hunger	Sleep	Discomfort	Accuracy
Hunger	178	2	6	0.9569
Sleep	4	120	5	0.9302
Discomfort	5	1	180	0.9677
Mean				0.9516

**Table 6:** Categorization accuracy for different genders.

	Correct	Incorrect	Total	Accuracy
Male	181	12	193	0.9378
Female	218	11	229	0.9519

**Table 7:** Comparison with other models.

No.	Reference	Method	Number of features	Validation	Dataset	Mean accuracy Hunger (%)	Mean accuracy Sleep (%)	Mean accuracy Discomfort (%)
1.	Hariharan et al. [33]	Extreme learning machine (ELM) kernel classifier	12	10-Fold cross-validation	Baby Chillanto database, Mexican Infants	90.23	—	81.98
2.	Liu et al. [34]	Compressed Sensing technique	1 (BFCC)	—	Neonatal intensive care unit (NICU) of a Hospital (anonymous).	68.42	68.42	70.64
			1 (LPC)	—		46.67	57.89	57.89
			1 (LPCC	—		48.89	47.37	62.67
			1 (MFCC)	—		53.33	68.42	71.05
3.	Saraswathy et al. [35]	Probabilistic neural network	17	10-Fold cross-validation	1. Baby Chillanto database, Mexican Infants 2. Hungarian deaf cry signals 3. Malaysian infant cry database (hospital Sultanah Bahiyah Alor Setar, Kedah, Malaysia)	—	—	90.79
		General regression neural network	17	10-Fold cross-validation	1. Baby Chillanto database, Mexican Infants 2. Hungarian deaf cry signals 3. Malaysian infant cry database (hospital Sultanah Bahiyah Alor Setar, Kedah, Malaysia)	—	—	78.71
4.	Orlandi et al. [26]	Logistic regression	22	10-Fold cross-validation	Infant cry dataset - S. Giovanni di Dio hospital, Firenze, Italy.	—	—	80.505
		Random Forest	22	10-Fold cross-validation	Infant cry dataset - S Giovanni di Dio hospital, Firenze, Italy.	—	—	86.702
	Alaie et al. [36]	Maximum a posteriori probability or Bayesian adaptation	2	Stratified K-fold cross-validation	Infant cry database - neonatology departments of several hospitals in Canada and Lebanon	—	—	65 .22
		Boosting mixture learning (BML) adaptation method for refining the mean and variance vectors.	2	Stratified K-fold cross-validation	Infant cry database - neonatology departments of several hospitals in Canada and Lebanon	—	—	67 .68
		Coupling old and boosting mixture learning adaptation estimates over the mean and variance vectors	2	Stratified K-fold cross-validation	Infant cry database - neonatology departments of several hospitals in Canada and Lebanon	—	—	68 .18
		Boosting mixture learning adaptation method for refining only the mean vectors	2	Stratified K-fold cross-validation	Infant cry database - neonatology departments of several hospitals in Canada and Lebanon	—	—	69 .59
6.	Jun et al. [37]	End-to-end deep Model using auto-encoder and K-means clustering	—	—	Real-world data collected using a sensor device.	—	—	97
7.	Parga et al. [38]	Cry-translation algorithm	10	—	ChatterBaby dataset	44	—	90.7
8.	Chang et al. [39]	DAG-SVM method	15	k-fold cross-validation	Infant cry dataset - national Taiwan university hospital Yunlin branch, Taiwan	86.36	76.81	95.45
9.	Proposed	Grouped-support-vector network	12	10-Fold cross-validation	Infant cry dataset - national Taiwan university hospital Yunlin branch, Taiwan	90.32	87.59	95.69

The article "An Efficient Classification of Neonates Cry Using Extreme Gradient Boosting-Assisted Grouped-Support-Vector Network" was published in 2021. Journal: J Healthc Eng.

## Data Availability

The original contributions generated for this study are included in the article; further inquiries can be directed to the corresponding author.
